The article "Ruxolitinib combined with vorinostat suppresses tumor growth and alters metabolic phenotype in hematological diseases" was published in 2017. Journal: Oncotarget.

# Ruxolitinib combined with vorinostat suppresses tumor growth and alters metabolic phenotype in hematological diseases

**DOI:** 10.18632/oncotarget.21951

**Published:** 2017-10-23

**Authors:** Monica Civallero, Maria Cosenza, Samantha Pozzi, Stefano Sacchi

**Affiliations:** ^1^ Department of Diagnostic, Clinical, and Public Health Medicine, University of Modena and Reggio Emilia, Modena, Italy

**Keywords:** ruxolitinib, vorinostat, apoptosis, metabolism, cancer therapy

## Abstract

JAK-2 dysregulation plays an important role as an oncogenic driver, and is thus a promising therapeutic target in hematological malignancies. Ruxolitinib is a pyrrolo[2.3-d]pyrimidine derivative with inhibitory activity against JAK1 and JAK2, moderate activity against TYK2, and minor activity against JAK3. Vorinostat is an HDAC inhibitor that reduces JAK-2 expression, thus affecting JAK-2 mRNA expression and increasing JAK-2 proteasomal deterioration. Here we hypothesized that the combination of ruxolitinib and vorinostat could have synergistic effects against hematological disease. We tested combinations of low doses of ruxolitinib and vorinostat in 12 cell lines, and observed highly synergistic cytotoxic action in six cell lines, which was maintained for up to 120 h in the presence of stromal cells. The sensitivity of the six cell lines may be explained by the broad effects of the drug combination, which can affect various targets. Treatment with the combination of ruxolitinib and vorinostat appeared to induce a possible reversal of the Warburg effect, with associated ROS production, apoptotic events, and growth inhibition. Decreased glucose metabolism may have markedly sensitized the six more susceptible cell lines to combined treatment. Therapeutic inhibition of the JAK/STAT pathway seems to offer substantial anti-tumor benefit, and combined therapy with ruxolitinib and vorinostat may represent a promising novel therapeutic modality for hematological neoplasms.

## INTRODUCTION

During hematopoietic ontogenesis, cytokines play key roles by initiating the intracellular signals that govern cell fate decisions, such as proliferation and differentiation. Most cytokine receptors lose intrinsic kinase activity and, therefore, often employ Janus kinase (JAK) as a signaling intermediate to facilitate downstream signaling. Receptor-related non-receptor tyrosine kinases, such as JAK1, JAK2, JAK3, and TYK2, are triggered after cytotoxic receptor activation [1]. JAK activation determines the phosphorylation of STAT transcription factors, including STAT1, STAT2, STAT3, STAT4, STAT5A, STAT5B, and STAT6. Following activation, STAT complexes translocate to the nucleus, bind DNA, and begin transcription [2, 3]. Dysregulation of JAK/STAT pathways can cause hematological illnesses and immunodeficiency disorders, and is implicated in the pathogenesis of some solid tumors [4]. Hematologic malignancies exhibit abnormal activation of JAK2 signaling [5]. The JAK2V617F mutation has been identified in different patients with neoplasms, supporting the development of JAK inhibitors to specifically target JAK signaling [6].

The article "Ruxolitinib combined with vorinostat suppresses tumor growth and alters metabolic phenotype in hematological diseases" was published in 2017. Journal: Oncotarget.

Ruxolitinib (INCB018424) is an orally administered, biologically available pyrrolo[2.3-d]pyrimidine derivative that shows inhibitory activity against JAK1 and JAK2, moderate activity against TYK2, and minor activity against JAK3 [7, 8]. Clinical trial results indicate a mechanism of action in which anti-JAK-STAT action mediates down-regulation of inflammatory cytokine activity [9, 10]. Ruxolitinib is approved by the US Food and Drug Administration (FDA) for use in myelofibrosis and polycythemia Vera, and is indicated for treatment of various solid tumors (breast, pancreatic, colorectal, head and neck, and prostate) and hematologic illnesses (CLL, ALL, AML, CML, and NSCLC) [11–14]. However, ruxolitinib does not appreciably reduce allele burden, and does not produce histologic or molecular cytogenetic remission in hematologic malignancies [15]. Furthermore, ruxolitinib resistance develops following chronic drug exposure [16], highlighting a clear need for combined therapies.

Histone deacetylase (HDAC) inhibitors are a promising group of therapeutic agents for various malignancies [17, 18]. Histone modifications may alter the expression and regulation of suppressor of cytokine signaling proteins (SOCS), a family of genes involved in JAK2-STAT3 signaling pathway inhibition [19, 20]. In October 2006, the FDA approved the HDAC inhibitor vorinostat for the treatment of advanced cutaneous T-cell lymphoma [21–23]. Most cancer treatments are intended to induce apoptosis through an extrinsic path or through a mitochondrial-intrinsic path via modulation of glucose metabolism [24]. Tumor cells show a surprisingly different metabolism compared to normal cells. The most important alteration is the Warburg effect [25, 26], which describes how tumor cells, even in the presence of abundant oxygen, continue to convert glucose to lactate with decreased mitochondrial respiration. Another important issue in cancer treatment is that hematologic cells strongly interact with the surrounding microenvironment, with bone marrow (BM) stroma potentially exerting protective effects from cytotoxic actions of drugs. In our present study, we screened the antitumor activity of ruxolitinib and vorinostat, each alone and in combination, in cell lines of hematologic malignancies including Hodgkin’s disease and selected subtypes of non-Hodgkin’s lymphoma, myeloma multiple, and chronic lymphatic leukemia. Our data suggested that all selected hematological malignancies were sensitive to ruxolitinib and vorinostat mono-therapy, but the combination of drugs synergistically increased the inhibitory effects, leading the tumor cells to undergo cessation of growth, differentiation inhibition, and increased apoptosis. We further co-cultured these 12 cell lines with mesenchymal cells, to examine how combined drug treatment competed with the protective effect exerted by the stroma. Finally, we examined metabolic aspects specifically the cellular depletion of ATP and lactate levels to better pinpoint a mechanism that could explain the effects of the drug combination. Our results suggested that the combination of ruxolitinib and vorinostat could affect proliferation by acting on the glycolytic and oxidative pathways. Since treatment with a combination of ruxolitinib and vorinostat showed a broad spectrum of action compared to individual drugs, such combined therapy may represent a promising new therapeutic modality for hematologic neoplasms.

The article "Ruxolitinib combined with vorinostat suppresses tumor growth and alters metabolic phenotype in hematological diseases" was published in 2017. Journal: Oncotarget.

## RESULTS

### Ruxolitinib interacts with vorinostat to induce cytotoxic effects in treated cell lines

First, we evaluated the cytotoxic effects (IC_50_) in the 12 hematological cell lines after 24 and 48 h of treatment with ruxolitinib and vorinostat as single agents. We used the MTT assay to quantify the inhibition of cell viability. In all cell lines, the IC_50_ of ruxolitinib ranged from 12–20 µM after 24 h of incubation, and from 1–5 µM after 48 h. The IC_50_ of vorinostat in all cell lines ranged from 15–25 µM after 24 h, and from 5–10 µM after 48 h.

To determine how viability was impacted by combined exposure to both ruxolitinib and vorinostat, we next incubated all cell lines for 24 and 48 h with both drugs at different concentration ratios, as indicated in the Chou-Talalay method, and again analyzed cell viability by MTT assay. We observed an additive effect (CI = 1) in the WSU-NHL, Granta 519, Jeko1, U266, HUT78, and L540 cell lines after 24 h of simultaneous exposure to ruxolitinib and vorinostat. In the remaining cell lines (RL, RPMI8266, Karpas422, Karpas299, MEC1, and L1236) the drug combination induced a synergistic effect (CI < 1) after 24 h. More specifically, the CI values ranged from 0.1–0.3, indicating strong synergy according to the Chou-Talalay theory (Figure 1). Notably, treatment with a combination of the two drugs at low concentrations for 48 h was too cytotoxic, causing obvious cell death revealed by exclusion assay with 0.2% Trypan Blue.

**Figure 1:** The antiproliferative activity of ruxolitinib and vorinostat, alone and in combination, after 24 h of treatment in all 12 cell lines Cell viability was evaluated by MTT assay. Results represent the mean ± standard error obtained from three independent experiments. To determine whether the combination of ruxolitinib with vorinostat was additive or synergistic, we investigated fixed ratios of combination of the drugs (R:V = 1:2), and applied isobologram analysis based on the Chou-Talalay method. Combination indices (CI) are reported in each graph.

The article "Ruxolitinib combined with vorinostat suppresses tumor growth and alters metabolic phenotype in hematological diseases" was published in 2017. Journal: Oncotarget.

### Combination of ruxolitinib and vorinostat exerts a synergistic cytotoxic effect on co-cultures of mesenchymal stem cell and tumor cell lines

Many studies support the theory that the bone marrow micro-environment can confer growth benefits and induce drug resistance in malignant cells [27, 28, 29]. Since we observed that different cell lines varied in their responses to the combination of ruxolitinib and vorinostat, we used a co-culture assay to investigate the possible protective effect of BM mesenchymal stem cells on the 12 cell lines. Ruxolitinib and vorinostat, alone and in combination, showed very weak cytotoxic effects (2–5%) after 24 h on all 12 cell lines in co-culture with hMSCs. This indicated defensive action of the BM microenvironment after 24 h of treatment. After 48 h, ruxolitinib-related cytotoxicity increased to 15–20% in all cell lines co-cultured with hMSCs, while treatment with vorinostat alone for 48 h induced a moderate decrease of cell viability (3–5%) in all 12 cell lines. After 48 h of co-culturing with ruxolitinib plus vorinostat, all cell lines showed an increase in cell death (45–55%), particularly the six more sensitive cell lines. After 72 h of co-culturing with both drugs, the six most sensitive cell lines did not show an increased percentage of viable cells, while the other cell lines continued to be protected by the microenvironment (Figure 2). The six more sensitive cell lines were cultured for 120 h, and the viability assay confirmed the prolonged synergistic effect of combined treatment with both drugs over the protective function of mesenchymal cells. Ruxolitinib and vorinostat, alone and in combination, exerted no cytotoxic effects on stromal cells alone from 24 to 120 h.

**Figure 2:** Viability of 12 cell lines *in vitro* when co-cultured with the stromal cell line hMSC for 24 to 72 h Tumor cells were harvested and stained with Trypan blue to determine cellular viability. Graphs indicate the viability index used to normalize the viability values to those under control conditions. Values are the mean ± standard error of three experiments. ^*^P < 0.001 Statistically significant differences *versus* control and single agents.

The article "Ruxolitinib combined with vorinostat suppresses tumor growth and alters metabolic phenotype in hematological diseases" was published in 2017. Journal: Oncotarget.

### Ruxolitinib and vorinostat, alone and in combination, regulate apoptosis via caspase activation and regulating anti-apoptotic proteins

To determine the apoptotic effects of ruxolitinib and vorinostat, alone and in combination, on all 12 cell lines, we evaluated the fraction of annexin V-positive cells (early and late apoptosis). After 24 h of single-drug treatment with ruxolitinib (5 µM) and vorinostat (10 µM), the percentage of apoptotic cells was not more than 5–10%. On the other hand, combined treatment with these drugs for 24 h led to an increase of the apoptotic fraction to 40–50% (Figure 3). Additionally, treatment of cells with ruxolitinib and vorinostat, alone and in combination, led to activation of caspase cleavage. Compared to single-agent treatment, combined treatment triggered substantially greater caspase-3 and caspase-8 activation in all 12 cell lines. Caspase-9 cleavage was detected only in the six more sensitive cell lines. To confirm whether ruxolitinib plus vorinostat caused caspase cascade, we treated all cell lines with the pan-caspase inhibitor z-VAD-fmk (10 µM) prior to combined drug treatment for 24 hrs. As shown in Figure 4, z-VAD-fmk remarkably restrained the cell apoptosis induced by ruxolitinib plus vorinostat in the sensitive cell line LH1236 and in the less sensitive cell line LH540. Comparable results were obtained in the other cell lines (data not shown).

**Figure 3:** Pro-apoptotic effects of ruxolitinib and vorinostat, alone and in combination Flow cytometric analysis revealed increased apoptosis after 24 h of combined treatment. ^*^P < 0.001 *versus* single-drug treatment.

**Figure 4:** Caspase activation triggered in 12 cell lines by exposure to ruxolitinib (5 µM) and vorinostat (10 µM), alone and in combination (ratio of 1:2) Caspase-8, caspase-9, and caspase 3 protease assays were used to assess the caspase proteolytic activity in lysates of cells following treatment with ruxolitinib and vorinostat, alone and in combination. The graph shows absorbance data obtained from treated RL cell lines. Co-exposure of cells to ruxolitinib and vorinostat led to markedly increased caspase activity in the six more sensitive cell lines.

To better clarify the apoptosis mechanism induced by ruxolitinib and vorinostat, we evaluated the expressions of some apoptosis-regulating proteins that induce programmed cell death (BAX, BID, and BAD), and of apoptosis inhibitors (BCL-2 and MCL-1). Expression levels were measured as mean fluorescence intensity (MFI) by flow cytometry after 24 h of incubation. In all cell lines, treatments with both single drugs and with the drug combination were associated with increased expressions of the BAX, BID, and BAD pro-apoptotic proteins. With regards to the anti-apoptotic proteins BCL-2 and MCL-1, the combination of ruxolitinib with vorinostat was associated with downregulation of both proteins in the six most sensitive cell lines, while single-drug treatment did not have this effect (Table 1).

The article "Ruxolitinib combined with vorinostat suppresses tumor growth and alters metabolic phenotype in hematological diseases" was published in 2017. Journal: Oncotarget.

**Table 1:** Expressions of apoptosis-regulating proteins that induce programmed cell death (BAX, BID, and BAD) and of apoptosis inhibitors (BCL-2 and MCL-1)

		RL	WSU	K422	HUT78	K299	MEC-1	L-540	L-1236	RPMI	U266	JEKO1	GRANTA
		N-fold increase/*decrease* in median MFI											
		(N-fold-proportion of protein expression (MFI) in examined sample vs untreated control, ns.-not significant)											
**BAX**	R	2,06	1,82	1,45	2	1,49	2,06	1,64	1,98	1,89	1,75	1,32	1,69
	V	2,11	1,8	1,54	1,6	1,63	2,13	1,601	1,92	1,85	1,7	1,28	1,72
	R+V	2,13	1,91	1,65	2,1	1,8	2,14	1,7	2,1	2,04	1,87	1,47	1,79
**BID**	R	1,89	1,71	0,84	1,84	2,13	2,04	1,42	2,1	2,001	1,86	1,6	1,79
	V	1,92	1,72	0,87	1,82	2,06	1,85	1,56	2	1,94	1,81	1,56	1,72
	R+V	1,94	1,84	1,09	1,87	2,4	2,32	1,63	1,9	2,05	2,1	1,64	1,89
**BAD**	R	1,69	1,52	1,35	1,89	1,52	1,63	1,64	1,36	2,05	1,91	1,2	1,32
	V	1,43	1,41	1,46	1,96	1,41	1,69	1,59	1,29	2,09	1,98	1,26	1,27
	R+V	1,64	1,49	1,35	2,13	1,74	1,98	1,84	2,1^*^	2,04	2,03	1,52	1,63
**BCL2**	R	0,91	0,35	1,2	0,89	0,91	2,3	1,56	1,54	2,1	0,38	1,06	0,95
	V	0,85	0,41	1,05	1,01	1,2	2,07	1,39	1,62	1,89	0,41	0,97	0,9
	R+V	0,26^*^	*0,24*	0,65^*^	0,65	0,35^*^	0,36^*^	0,76^*^	0,37^*^	0,51^*^	*0,32*	0,98	0,74
**MCL-1**	R	1,93	0,63	2,1	0,69	2,23	1,32		0,95	1,89	1,58	1,15	0,84
	V	1,72	0,59	2,13	0,99	2	1,09	0,95	1,04	2,14	1,46	0,98	0,53
	R+V	0,84^*^	*0,59*	0,48^*^	*0,54*	0,61^*^	0,37^*^	0,74	0,29^*^	0,54^*^	0,67^*^	0,78	0,55
		^*^statistically significant differences vs control											

Expression levels were measured as mean fluorescence intensity (MFI) by flow cytometry after 24 h of incubation with ruxolitinib plus vorinostat. Data are the mean of three different experiments. ^*^P < 0.001 Statistically significant differences versus control and single agents.

### The combination of ruxolitinib and vorinostat influences the cell cycle and related proteins

In all 12 cell lines, ruxolitinib and vorinostat treatment alone did not significantly affect the cell cycle distribution. On the other hand, the combination treatment induced cell cycle progression defects, with a marked increase of G2-M arrest after 24 h. Compared to single-agent treatment, cells subjected to combined treatment with ruxolitinib and vorinostat showed a slight decrease of cells in S phase and sub G0/G1 phase, and a significantly decreased percentage of cells in G0/G1 (Figure 5A and 5B). To investigate the effects of ruxolitinib and vorinostat on cell cycle-related proteins, we evaluated the expressions of AURORA A, CCND1, p27, and p21 in all 12 cell lines. Combination drug treatment induced upregulated expression of the CDK inhibitors p21 and p27, and downregulated expression of the positive regulators of cell cycle progression AURORA A and CCND1 (Figure 5C–5E). The results of densitometric semi-quantification of western blot bands were normalized by total proteins to the untreated control levels of p27, p21, AURORA A, and CCND1. Figure 5 presents the effects of combined treatments in the RL cell line. This cell line was randomly chosen for display, and the results obtained in the RL cell line are comparable with the other 11 cell lines.

The article "Ruxolitinib combined with vorinostat suppresses tumor growth and alters metabolic phenotype in hematological diseases" was published in 2017. Journal: Oncotarget.

**Figure 5:** Treatment with ruxolitinib plus vorinostat influences the cell cycle and related proteins (**A**) Representative flow cytometry histograms of the cell cycle distribution of the RL cell line. M1 indicates sub-G0/g1; M2, G0/G1; M3, S; and M4, G2/M. (**B**) Cell cycle profile of RL cells treated for 24 h with ruxolitinib (5 µM) and vorinostat (10 µM), alone and in combination (ratio, 1:2). Bars represents the mean ± standard error estimated based on the rate of cells in the following cell cycle fraction: sub-G1, G0-G1, S, and G2-M. ^*^p < 0.001 Statistically significant differences *versus* control and single agents. (**C**–**E**) Western blot of cellular extracts from RL cell line. The levels of p21, p27, AURORA A, and CCND1 were analyzed using Quantiti One software (Bio-Rad Laboratories) and expressed as relative value compared to total proteins. ^*^p < 0.001 Statistically significant differences *versus* control and single agents.

### Combination of ruxolitinib and vorinostat enhances dephosphorylation of proteins of the JAK-STAT pathways

In all 12 cell lines, we tested the ability of ruxolitinib and vorinostat, alone and in combination, to inhibit some JAK family members. Without treatment, all cell lines expressed comparable levels of total JAK2, p-JAK2, total STAT3, p-STAT3, total STAT5, and p-STAT5 proteins (Figure 6A). Following 24 h of treatment with ruxolitinib (5 µM), we found diminished p-JAK2 expression in the RL, RPMI8266, and Karpas299 cell lines. All cell lines showed diminished expressions of the p-STAT3 and p-STAT5 proteins, as can be observed from the densitometric analysis reported in Figure 6B. Vorinostat treatment alone did not significantly alter p-JAK2 expression in any cell line, and slightly impacted the expressions of p-STAT3 and p-STAT5 in all cell lines (Figure 6C). Finally, 24 h of treatment with the combination of ruxolitinib and vorinostat (ratio = 1:2) caused marked suppressive effects on the expressions of p-JAK2, p-STAT3, and p-STAT5 in all cell lines (Figure 6D).

The article "Ruxolitinib combined with vorinostat suppresses tumor growth and alters metabolic phenotype in hematological diseases" was published in 2017. Journal: Oncotarget.

**Figure 6:** Western blot analysis of JAK2-STAT3-5 pathway protein levels in cell lines after 24 h of treatment with ruxolitinib (5 µM) and vorinostat (10 µM), alone and in combination (ratio, 1:2) Whole-cell lysates from cell lines no treated, treated with Ruxolitinib, with Vorinostat and with the combination were subjected to protein gel blotting using the indicated antibodies (**A**–**F**). Densitometric semi-quantification of bands normalized to the untreated control is shown below the immunoblot bands. The samples come from the same experiment and that the gels / blots have been treated in parallel. In the cell lines not shown in the figure we obtained blots comparable.

### Ruxolitinib and vorinostat influence secretion of IL-10, IL-6, and IL-17A

JAK-STAT pathways are activated through tyrosine phosphorylation of the cytoplasmic domains of cytokine receptors upon cytokine binding. In particular, IL-6, IL-10, and IL-17A signaling occurs through both JAK1 and JAK2 [30–32]. We evaluated the expressions of IL-6, IL-10, and IL-17A in all 12 cell lines relative to control. After 24 h of treatment with the combination of ruxolitinib and vorinostat, all 12 cell lines showed significantly decreased (*P* < 0.001) secretion of IL-10 into the media (Figure 7A). Moreover, all 12 cell lines showed similar decreases in IL-6 secretion after treatment with ruxolitinib and vorinostat, both alone and in combination (Figure 7B). Interestingly, combination drug treatment particularly inhibited sustained production of IL-17A in the six more sensitive cell lines (Figure 7C).

**Figure 7:** Secretion of IL-10, IL-6, and IL-17A after treatment with ruxolitinib and vorinostat Cells were stimulated with ruxolitinib (5 µM) and vorinostat (10 µM), alone and in combination (ratio, 1:2), and a multiplex assay was used to determine the levels of IL-10, IL-6, and IL-17A secreted into the media. In all graphs, error bars represent the standard error of three independent experiments. ^*^P < 0.001 *versus* control and single agents.

### Ruxolitinib and vorinostat affect autophagy

Autophagy plays a complex and often contradictory role in tumor progression, and is a promising target for cancer treatment [33]. To study autophagy, we quantified the p62 protein response in all 12 cell lines following treatment with ruxolitinib and vorinostat, alone and in combination. Quantitative determination of p62 revealed that treatment with a combination of ruxolitinib and vorinostat induced autophagy comparable to that observed in cells subjected to 12 h of serum starvation. Combined treatment with the two drugs along with the autophagy inhibitor chloroquine inhibited autophagic flux of cancer (Figure 8). In the same cellular lysate used to study autophagy, we also evaluated cellular apoptosis (data not shown). The results suggest that the combination of ruxolitinib and vorinostat induced both apoptosis and autophagy.

The article "Ruxolitinib combined with vorinostat suppresses tumor growth and alters metabolic phenotype in hematological diseases" was published in 2017. Journal: Oncotarget.

**Figure 8:** Quantitative determination of p-62 expression in all 12 cell lines after treatment for 24 h with ruxolitinib (5 µM) and vorinostat (10 µM), alone and in combination Results represent the mean ± standard error of three independent experiments.

### Exposure to the ruxolitinib and vorinostat combination triggers ROS generation

We previously found that the combination of ruxolitinib and vorinostat triggers the mitochondria-mediated signaling pathway. Alterations in the redox state of apoptotic cells could be related to activation of the final stage of the caspase cascade [34, 35]. ROS generation could play an important role in cytotoxicity induced by ruxolitinib and vorinostat. Thus, we investigated the effects of these drugs, both alone and in combination, with co-administration of N-acetyl cysteine (NAC) antioxidants to block ROS generation. Single-agent administration of ruxolitinib or vorinostat exerted only a slight-to-moderate effect on ROS generation in all 12 cell lines (Figure 9). Combined drug treatment resulted in a moderate increase of ROS generation in the WSU and U266 cell lines—about 1.5-fold higher than the untreated controls. Moreover, combined drug treatment induced a significant (*P* < 0.001) increase of ROS production in the six more sensitive cell lines. Co-treatment with NAC effectively blocked ROS generation in all 12 cell lines.

**Figure 9:** Treatment with ruxolitinib and vorinostat, alone and in combination, affects ROS generation ROS levels were determined by flow cytometry, and histograms show quantitative analysis of ROS generation. Increased ROS levels were observed in the six more sensitive cell lines after combined drug treatment for 24 h. Co-administration of the antioxidant N-acetyl cysteine NAC blocked the increase of ROS generation. Results represent the mean ± standard error obtained from three independent experiments. ^*^P < 0.001.

### Combined treatment with ruxolitinib and vorinostat decreased ATP generation, lactate levels and GLUT1 expression

Highly proliferative cells, such as cancer cells, are characterized by alterations in energy metabolism, including increased anaerobic glycolysis [36]. We initially measured the amount of ATP in culture medium after cell lines were incubated for 24 h with ruxolitinib (5 µM) and vorinostat (10 µM), alone and in combination. We observed a decreased glycolytic rate in the six more sensitive cell lines following treatment with ruxolitinib plus vorinostat (Figure 10). Addition of the mitochondrial ATP synthase inhibitor oligomycin led to an increased glycolytic rate in both treated and untreated cell lines. We also monitored the amount of lactate released in all 12 cell lines. The six more sensitive cell lines showed decreased lactate production after incubation with ruxolitinib combined with vorinostat (Figure 11). Lactate production can vary in accordance with any alteration of the glycol pathway; however, our experiments were performed in an *in vitro* model with cultured cells, thus limiting fluctuations in lactate levels. Based on our results, we further examined whether cells treated with the combined drugs would show decreased expression of GLUT1, the key enzyme of the glycolytic pathway. After 24 h of incubation with ruxolitinib plus vorinostat, we detected decreased GLUT1 expression in all 12 cell lines, with no significant difference between the most sensitive cell lines and the remaining cell lines (Figure 12).

The article "Ruxolitinib combined with vorinostat suppresses tumor growth and alters metabolic phenotype in hematological diseases" was published in 2017. Journal: Oncotarget.

**Figure 10:** Intracellular ATP levels in response to ruxolitinib and vorinostat treatment Intracellular ATP levels were measured in control and drug-treated cells after 24 h. ATP levels are expressed as % of untreated control. Data represent mean ± standard error of three independent experiments.

**Figure 11:** Lactate levels after treatment with ruxolitinib (5 µM) and vorinostat (10 µM), alone and in combination Cells were cultures with drugs (alone and in combination) for 24 h. Then the supernatant was collected and lactate levels were determined by colorimetric analysis. Data represent mean ± standard deviation of three independent experiments. ^*^p < 0.001 Statistically significant differences *versus* control and single agents.

**Figure 12:** GLUT1 protein levels in all 12 cell lines after treatment with ruxolitinib plus vorinostat for 24 h Densitometric semi-quantification of bands normalized to the untreated control is shown below the immunoblot bands.

## DISCUSSION

JAK-2 dysregulation plays an important role as an oncogenic driver, prompting increasing interest in JAK-2 inhibitors for therapy against hematological malignancies [37, 38]. The translation of first-generation JAK inhibitors (tofacinib, oclacitinib, baricitinib, and ruxolitinib) to clinical application in myelofibrosis represents a substantial advance in patient treatment (ClinicalTrials.gov, U.S. National Institutes of Health, Bethesda, MD, USA: http://clinicaltrials.gov/). The success of ruxolitinib has inspired the rapid development of additional JAK inhibitors, extending the armamentarium for targeted therapy of malignancies driven by JAK signaling [39]. However, the curative potential of JAK inhibitors appears to be limited, and the survival benefits are controversial with limited follow-up available [40]. Since JAK-2 plays an essential role hematopoiesis, JAK-2 inhibition is associated with hematologic toxicities that limit dose escalation, which may in turn limit the extent of target inhibition. HDAC inhibitors reduce JAK-2 expression, likely due to effects on JAK-2 mRNA expression and through increased JAK-2 proteasomal deterioration [41–43]. Combination therapy might prove beneficial due to synergistic impacts on oncogenic transformation, could enable the effective use of lower doses of the different agents with better tolerability, and might avoid or delay the development of drug resistance.

The article "Ruxolitinib combined with vorinostat suppresses tumor growth and alters metabolic phenotype in hematological diseases" was published in 2017. Journal: Oncotarget.

Our present results show that combination treatment with ruxolitinib and vorinostat had improved effects on proliferation and apoptosis in an *in vitro* model of hematological disease. We found that a combination of the two drugs showed greater efficacy compared to low-dose single-agent treatment with ruxolitinib and vorinostat in 12 cell lines, including two B-cell lymphomas, two T lymphoma, one chronic B-cell leukemia, two myeloma multiple, two Hodgkin lymphoma, two mantle lymphoma, one non-Hodgkin lymphoma. The results of combination treatment were additive in both mantle cell lymphoma cell lines, in one LH cell line, in one myeloma cell line, in one T-cell lymphoma cell line, and in one B-cell lymphoma cell line. In the remaining cell lines, the combination of the two drugs had highly synergistic effects. These results led us to postulate that this combination may have the potential to overcome protective effects of a tumor microenvironment. Indeed, tumor cells treated with the combination of ruxolitinib and vorinostat for 48 h were not protected by co-culture with stromal cells. The synergistic cytotoxic action of this drug combination was maintained for up to 120 h. We also found that the ruxolitinib and vorinostat combination influenced the cell cycle distribution, increasing G2-M phase arrest after 24 h in all 12 cell lines. Correspondingly, the combined treatment affected the related cell cycle proteins. In all 12 cell lines, treatment with ruxolitinib and vorinostat for 24 h resulted in upregulation of the cell cycle regulators p21 and p27, and downregulation of CCND1 and AURORA A, which are important in regulating the cell cycle control points. These results confirmed that this combination of drugs induced tumor growth inhibition.

After 24 h of single-agent treatment with ruxolitinib or vorinostat, less than 10% of cells were apoptotic annexin V-positive cells. However, this proportion of apoptotic cells increased to 50% in all 12 cell lines after treatment with ruxolitinib combined with vorinostat. Caspases play a very important role in programmed cell death and are thus attractive targets for the development of new cancer therapies. We chose to study the caspase initiator caspase-8, and the caspase effectors caspase-9 and caspase-3. After 24 of combined drug treatment, we detected cleavage of caspase-8 and caspase-3 in all 12 cell lines, suggesting activation of the extrinsic apoptotic pathway. Moreover, only the six most sensitive cell lines showed increases in the cleaved form of caspase-9, suggesting caspase activation of mitochondrial events regulating intrinsic apoptosis. The most sensitive cell lines also differed from the other cell lines in terms of the regulation of anti-apoptotic proteins. After treatment with the drug combination, all 12 cell lines showed increased expression of the pro-apoptotic proteins BAX, BID and BAD, but only the six more sensitive cell lines showed downregulation of the apoptotic inhibitors BCL-2 and MCL-1. These results confirmed the possibility that ruxolitinib combined with vorinostat may differentially target signaling pathways in the six more sensitive cell lines.

The article "Ruxolitinib combined with vorinostat suppresses tumor growth and alters metabolic phenotype in hematological diseases" was published in 2017. Journal: Oncotarget.

JAK/STAT activation has been demonstrated in hematological malignancies, providing the rationale for various therapeutic approaches involving JAK kinase inhibitors [44–46]. Here we assessed JAK/STAT activation based on the expressions of phospho-JAK2, STAT3, and STAT5. Notably, the combination of ruxolitinib and vorinostat increased the de-phosphorylation of JAK2, STAT3, and STAT5, blocking the pathway. This may be partly due to ruxolitinib’s inhibitory effect on JAK2, but may also be influenced by the fact that vorinostat targets the JAK pathway. It has been reported that when cells become resistant to JAK2 inhibitors, they remain dependent on the expression of JAK2 proteins; thus, our present findings may suggest alternative therapy that indirectly degrades JAK2 [47]. JAK/STAT activation is closely related to binding of cytokines to their receptors. Tumors contain high numbers of circulating cytokines, making them attractive as potential therapeutic targets. Binding of IL-6, IL-10, and IL-17 to their receptors promotes the activation of JAKs [48, 49]; however, the anti-tumor immunomodulatory role of IL-6, IL-10 and IL-17 remains unclear and appears contradictory in some aspects. All three interleukins are released into healthy tissues, as well as into many tumor infiltrates in larger quantities. The ability of interleukins to provide access to tissues and to recruit large numbers of immune cells has obvious advantages for antitumor responses, especially in solid tumors. However, cytokines that facilitate immune cell access to cancers may also generate conditions that facilitate tumor cell migration and diffusion via circulation [50]. Our present experiments showed that ruxolitinib combined with vorinostat reduced IL-10 and IL-6 secretion comparably among all 12 cell lines. On the other hand, IL-17A expression was only significantly reduced after combined treatment in the six more sensitive cell lines. These results suggest that the drug combination had a broad range of effects that acted upstream of JAK/STAT pathway inhibition.

The article "Ruxolitinib combined with vorinostat suppresses tumor growth and alters metabolic phenotype in hematological diseases" was published in 2017. Journal: Oncotarget.

JAK is reportedly involved in autophagy induction for immune regulation in various cancer cells [51–52]. Thus, we investigated the cross-talk between the JAK pathway and the autophagy process in our treated cell lines. We showed that ruxolitinib and vorinostat, alone and in combination, induced a decrease of the amount of the autophagy-related p62 protein in cancer cells, indicating activation of the autophagic system. Autophagy and apoptosis are mechanisms that cause increased oxidative stress, leading to ROS production. Increased ROS production is detected in various cancers, and reportedly plays several roles linked to pro-tumorigenic signaling, as well as roles related to anti-tumorigenic signaling, initiating oxidative stress-induced tumor cell death [55]. Our present results indicated that ruxolitinib and vorinostat synergistically induced apoptosis in the six more sensitive cell lines, associated with markedly increased ROS generation. Co-administration of the ROS scavenger LNAC reduced the increased ROS levels induced by the ruxolitinib and vorinostat combination. These results could be very interesting considering that tumor cells have an altered redox balance compared to their normal counterparts, which identifies ROS manipulation as a potential target for cancer therapies. Cancer cells exhibit increased rates of aerobic glycolysis, and the modulation of glucose metabolism reportedly affects intrinsic and extrinsic apoptosis. Our data show that combined treatment with ruxolitinib plus vorinostat altered tumor cell metabolism by reducing the glycolic state, lead to the greater sensitivity of the six cell lines.

In conclusion, here we show that treatment with a combination of ruxolitinib and vorinostat led to decreased glucose metabolism, and that this partial reversion of the Warburg effect was associated with ROS production, apoptosis, and cell growth inhibition. Testing these drugs under different cell culture conditions provided information regarding drug efficacy, and could help predict pharmacological effects that may be difficult to translate from *in vitro* and *ex vivo* conditions to clinical practice. Our present results offer evidence of synergistic interaction between ruxolitinib and vorinostat in hematological tumor cells, and provide the rationale to support clinical studies using the combination of both agents in patients.

The article "Ruxolitinib combined with vorinostat suppresses tumor growth and alters metabolic phenotype in hematological diseases" was published in 2017. Journal: Oncotarget.

## MATERIALS AND METHODS

### Cell lines

We purchased the mantle cell lymphoma cell lines GRANTA519 and Jeko1, multiple myeloma cell lines U266 and RPMI8266, B-cell lymphoma cell lines Karpas422 and RL, cutaneous T-cell lymphoma cell line HUT78, anaplastic cell lymphoma cell line Karpas 299, chronic B-cell leukemia cell line MEC1, and Hodgkin lymphoma cell lines LH540 and LH1236 from Deutsche Sammlung von Mikroorganismen und Zellkulturen GmbH. Cell line characteristics are available online (http://www.dsmz.de/human_and_animal_cell_lines/main). The B-cell lymphoma cell line WSU-NHL was kindly provided by Dr. M. Introna (Bergamo, Italia). GRANTA519 and MEC1 cells were cultured in Iscove’s MEM supplemented with 10% fetal bovine serum (FBS), 2 mM L-glutamine, penicillin (100 U/mL), and streptomycin (100 U/mL). All other cell lines were cultured in RPMI-1640 supplemented with 10% fetal bovine serum (FBS), 2 mM L-glutamine, penicillin (100 U/mL), and streptomycin (100 U/mL) (all purchased from Euroclone). The human mesenchymal stem cells (hMSC) were purchased from Tebu Bio and cultured in complete MSC expansion media (Tebu Bio). Cells in the logarithmic growth phase were used for experiments.

### Drugs

Ruxolinostat and vorinostat were purchased from Selleck Chemicals. Each was dissolved in dimethylsulfoxide (DMSO; Euroclone) to create 10^−2^ M stock solutions that were stored at −80°C. These stock solutions were further diluted using cell culture medium to the appropriate concentrations for use. Oligomycin was purchased from Sigma Aldrich.

### Assessment of cell viability and proliferation

In dose-response experiments, cell lines were treated with increasing concentrations of ruxolitinib and vorinostat for 24 and 48 h. Relative viable cells were determined by MTT assay (cellTiter non-radioactive cell proliferation assay; Promega). The absorbance at 550 nm was measured using an ELISA reader. We determined the drug concentration required for 50% inhibition of cell proliferation (IC_50_) using Calcusyn software (Biosoft, Cambridge, UK) applying the median-effect method. Viability was assessed by exclusion assay with 0.2% Trypan Blue (Euroclone). DMSO was directly added to control samples and used as a drug solvent for drug-treated samples, and the DMSO concentration was kept constant (0.1%) among treatments for all experiments. The maximum final concentration of DMSO (< 0.1%) did not affect cell proliferation and did not induce cytotoxicity in the tested cell lines.

The article "Ruxolitinib combined with vorinostat suppresses tumor growth and alters metabolic phenotype in hematological diseases" was published in 2017. Journal: Oncotarget.

### Combination study

To investigate the inhibitory effects of drug combination treatment, we used isobologram analysis, following the Chou-Talalay method that provides algorithms for automated computer simulation of synergism and/or antagonism based on the median-effect equation derived from the mass action law [53, 54]. We used CalcuSyn Windows software for dose-effect analysis and synergism/antagonism quantification (Biosoft, Cambridge, United Kingdom). The evaluation of drug synergism based on a median-effect equation is commonly described in the literature [55]. A combination index (CI) of > 1 indicates antagonism, a CI of 1 denotes additivity, and a CI of < 1 indicates synergism. More specifically, CI values ranging from 0.1–0.3 are considered to indicate strong synergism, 0.3–0.7 synergism, and 0.7–0.85 moderate synergism.

### Co-culture of cell lines with bone marrow stromal cells

Human mesenchymal stem cells hMSC cells were cultured following the recommended protocol. Mesenchymal cells were seeded in triplicate in 96-well plates, and incubated for 48 h to reach confluence. Once the 12 cell lines adhered to the CM stroma, the co-cultures were treated with ruxolitinib and vorinostat, alone or in combination. After 24, 48, 72, 96, and 120 h, the cells were harvested and assessed for viability.

### Cytometric analysis for apoptosis

To determine the apoptosis rate after 24 and 48 hours of drug exposure, we performed flow cytometry using the Annexin V/Propidium Iodide Staining kit (Miltenyi Biotec, Germany), following the manufacturer’s instructions. At least 20,000 events were acquired using a FACSCalibur cytometer (Becton Dickinson, San Jose, CA, USA), which were then analyzed using FlowJo Software (Tree Star, Ashland, OR, USA).

In preparation for intracellular marker staining, the cells were washed with 1% v/v FBS-PBS (staining buffer), fixed in 4% w/v paraformaldehyde (20 min at 4°C), and permeabilized with 0.1% saponin in PBS. Then the cells were incubated for 1 h at 4°C with primary antibodies against p-BAD (Ser112), BID, BAX, MCL-1 and BCL-2 (all from Cell Signaling). Finally, the cells were incubated with fluorophore-tagged secondary antibodies for 45 min at 4°C, and the cells were analyzed using a FACSCalibur flow cytometer. The results were analyzed using the CellQuest program. Whenever possible, the immunophenotype results were expressed as the percentage of positive cells.

We measured caspase-3, caspase-8, and caspase 9 activity using colorimetric assay kits purchased from Enzo Life Sciences, in accordance with the manufacturer’s instructions. Samples were analyzed using an ELISA reader.

The article "Ruxolitinib combined with vorinostat suppresses tumor growth and alters metabolic phenotype in hematological diseases" was published in 2017. Journal: Oncotarget.

### Cell cycle analysis

For cell cycle distribution analysis, cells were harvested after 24 h of drug treatment. These cells were fixed in ethanol (95%) containing RNase (10 g/mL), stained for 15 min with propidium iodide (PI, 50 m/mL), and then analyzed with a FACSCalibur cytometer. We calculated the percentages of cells in the subG1/G0 (dead cells), G1/G0, S, and G2/M phases of the cell cycle (determined in relation to DNA histogram analysis) using Modifit LT software (Verity Software House, Topshem, ME, USA).

### Autophagy detection

We quantified autophagy in cell lysates using the quantitative immunometric detection method provided by the p62 (sequestosome 1) ELISA kit (Enzo Life Science, Farmingdale, NY, USA) following the manufacturer’s instructions.

### Measurement of reactive oxygen species (ROS) production

Reactive oxygen species (ROS) production was analyzed by incubating cells with 2′,7′-dicholorodihydrofluorescein diacetate (DCFH-DA; Sigma Aldrich) in complete medium for 30 minutes at 37°C. Fluorescence was quantified with a FACSCalibur cytometer (Becton Dickinson), and these data were analyzed using FlowJo Software (Tree Star).

### Lactate and ATP assay

We measured lactate and ATP levels using an L-lactate assay colorimetric kit and an ATP assay colorimetric kit (Abcam), following the manufacturer’s instructions. In the L-lactate assay kit, lactate is oxidized by lactate dehydrogenase to generate a product that interacts with a probe, producing a color (OD = 450 nm). The ATP assay kit is based on the phosphorylation of glycerol, generating a product that can be colorimetrically quantified (OD = 570 nm).

### Western blot analysis

After drug treatments, 1 × 10^6^ cells were pelleted and then lysed using the Mammalian Cell Extraction Kit (BioVision, Milpitas, CA, USA) following the manufacturer’s instructions. Proteins (100 µg/lane) were electrophoresed on 4–20% (w/v) Miniprotean TGX Precast Gels (Bio-Rad, USA), and then transferred to nitrocellulose membranes (Bio-Rad Laboratories, Hercules, CA, USA). Membranes were immunoblotted using the following primary antibodies: total JAK2, p-JAK2, total STAT3, p-STAT3, total STAT5, p-STAT5, CCND1, AURORA A, p21, p27 and GLUT-1. Next, the membranes were incubated with species-specific horseradish peroxidase (HRP)-conjugated secondary antibody. All above-mentioned antibodies were purchased from Euroclone. Blots were developed using SuperSignal West Pico Chemiluminescent Substrate (Thermo Scientific, Rockford, IL, USA), and images were acquired using Chemidoc XRS+ and analyzed with Image Lab Software v.3.0 (Bio-Rad Laboratories).

The article "Ruxolitinib combined with vorinostat suppresses tumor growth and alters metabolic phenotype in hematological diseases" was published in 2017. Journal: Oncotarget.

### Measurement of IL-6, IL-10, and IL-17a in cell culture supernatants

Cells were cultured at a density of 5 × 10^5^ cells/mL for 24 h with ruxolitinib and vorinostat, alone and in combination. Then the supernatants were collected and analyzed for levels of the cytokines IL-6, IL-10, and IL-17a using a Human Magnetic Luminex Assay (R&D Systems), following the manufacturer’s instructions.

### Statistical analysis

All experiments were independently repeated three times, with multiple replicates within each run. Data are expressed as mean ± standard error. We analyzed statistical differences between control and drug-treated cells using one-way ANOVA, and *P* values less than .05 were assigned significance. Data were analyzed using the Stata 8.2/SE package (StataCorp LP, College Station, TX, USA).
